# Sliding Mode Control of Flexible Articulated Manipulator Based on Robust Observer

**DOI:** 10.1155/2022/2440770

**Published:** 2022-01-04

**Authors:** Yanghua Gao, Hailiang Lu

**Affiliations:** Information Center, China Tobacco Zhejiang Industrial Co., Ltd, Hangzhou 310008, China

## Abstract

In this paper, a robust observer-based sliding mode control algorithm is proposed to address the modelling and measurement inaccuracies, load variations, and external disturbances of flexible articulated manipulators. Firstly, a sliding mode observer was designed with exponential convergence to observe system state accurately and to overcome the measuring difficulty of the state variables, unmeasurable quantities, and external disturbances. Next, a robust sliding mode controller was developed based on the observer, such that the output error of the system converges to zero in finite time. In this way, the whole system achieves asymptotic stability. Finally, the convergence conditions of the observer were theoretically analyzed to verify the convergence of the proposed algorithm, and simulation was carried out to confirm the effectiveness of the proposed method.

## 1. Introduction

Flexible manipulators are increasingly applied in industrial and aerospace fields, such as welding robots, industrial production lines, mechanical arms of aircraft, and so on, owing to their energy efficiency, high speed, and low contact impact. More and more attention has been paid to the research of flexible manipulators, along with the development of aerospace technology, robotics, marine engineering, and industrial engineering. Flexible manipulators are now extensively used to comfort humans in different areas of work, which involves risky and tedious works such as painting, cutting, dispensing, material handling, machine tending, machining, and assembly. However, each flexible manipulator is an extremely complex, dynamic system with highly nonlinear, strongly coupled, and time-varying features. The system behaviors are complex and dynamic due to load variations, uncertain external perturbations, and inherent vibrations [1–3]. Hence, flexible manipulators can hardly be modelled or measured accurately, calling for a well-designed controller [4–8]. Against this backdrop, it is theoretically and practically significant to explore the response speed and control accuracy of trajectory tracking for the double-linked flexible-joint manipulator [9].

To address the above problems, Lee et al. [10] designed an adaptive proportional-derivative (PD) controller to improve the trajectory tracking accuracy of the flexible-joint manipulator but did not consider the stability of the manipulator system. Lee and Lee [11] proposed a hybrid control strategy to optimize the design of the controller and generate hybrid trajectories. The strategy enhances the robustness of the flexible-joint manipulator system, yet it failed to take into account the trajectory tracking accuracy of the manipulator. Dong et al. [12] presented a fuzzy optimal control method for the design of a robust adaptive controller and demonstrated that the method ensures accurate and robust trajectory tracking of the flexible-joint manipulator. However, the manipulator's response speed of trajectory tracking was not taken into consideration. Abd Latip et al. [13] automatically adjusted the control gain online with an adaptive proportional-integral-derivative (PID) controller, which supports the control of the single-link flexible manipulator even after the actuator failure.

Ahanda et al. [14] addressed the robust adaptive control of a robotic manipulator under uncertain dynamics and joint space constraints and adopted command filters to overcome the time derivatives of virtual control, eliminating the need for differentiating the desired trajectory. In addition, a barrier Lyapunov function was introduced to handle joint space constraints, and a robust adaptive support vector regression architecture was employed to suppress filtering errors, approximation errors, and dynamic uncertainties. Based on unknown input observer (UIO), Wang et al. [15] put forward a novel funnel nonsingular terminal sliding mode control (FNTSMC) method for servomechanisms with unknown dynamics, e.g., nonlinear friction, uncertainties, and external disturbances. He et al. [16] created a full-state feedback neural network (NN) control to mitigate the uncertainties and enhance the robustness of the dynamic system of a flexible-joint manipulator. Through a Lyapunov stability analysis, it was demonstrated that the controller can ensure the stability of the flexible-joint manipulator system and guarantee the boundedness of system state variables, by choosing appropriate control gains. Rahmani and Belkheiri [17] came up with a novel approach for adaptive control of flexible multilink robots in the joint space, proved that the approach is valid for a class of highly uncertain systems with arbitrary but bounded dimensions, and realized trajectory tracking by developing a stable inversion for robot dynamics using only joint angle measurements. Guo et al. [18] investigated the repetitive motion planning (RMP) of robotic manipulators under the high precision of joint angle repeatability and end-effector motion and applied a special difference rule to discretize the existing RMP scheme with *P*-based formulation, yielding a novel pseudoinverse-based (*P*-based) RMP scheme for robotic manipulators.

Through the above analysis, this paper proposes a sliding mode control strategy based on the robust observer. Firstly, a sliding mode robust observer was designed in light of the unmeasurable state, the modelling uncertainty, and the external disturbance moment of the flexible-joint manipulator. Next, a sliding mode controller was designed to track the positions of the first and second joints of the manipulator, aiming to realize the finite-time control of the system. Meanwhile, the convergence of the observer and controller was analyzed to present the convergence conditions. Finally, the effectiveness of the proposed method was verified through simulation.

## 2. Problem Description

The dynamics of the flexible-joint manipulator can be expressed as

(1) $$\begin{array}{c} \left\{\begin{array}{c} I\ddot{\theta }+K\left(\theta -\theta_{m}\right)+Mgl\;\sin\;q=0,\\ J{\ddot{\theta }}_{m}-K\left(\theta -\theta_{m}\right)=u, \end{array}\right) \end{array}$$

where *θ* and *θ*_*m*_ are the angular positions of the link and rotor, respectively; *I* and *J* represent the rotational inertia of the link and rotor, respectively; *K* is the joint stiffness coefficient; *M*, *g*, and *l* are the link mass, gravitational acceleration at the link's center of gravity, and joint length, respectively; and *u* is the motor torque input.

Let *x*_1_=*θ*, $x_{2}=\dot{\theta }$, *x*_3_=*θ*_*m*_, and $x_{4}={\dot{\theta }}_{m}$ be state variables. Considering modelling uncertainty and external disturbance moments, the underdriven form of equation (1) can be obtained as

(2) $$\begin{array}{c} \left\{\begin{array}{c} {\dot{x}}_{1}=x_{2},\\ {\dot{x}}_{2}=a_{1}x_{3}+f_{1}\left(x_{1}\right)+\Delta_{1}\left(t\right),\\ {\dot{x}}_{3}=x_{4},\\ {\dot{x}}_{4}=a_{2}u+f_{2}\left(x_{1},x_{3}\right)+\Delta_{2}\left(t\right), \end{array}\right) \end{array}$$

where *a*_1_=(*K*/*I*); *f*_1_(*x*_1_)=−(*Mgl*/*I*) · sin  *x*_1_ − (*K*/*I*) · *x*_1_; *a*_2_=(1/*J*); *f*_2_(*x*_1_, *x*_3_)=(*K*/*J*) · (*x*_1_ − *x*_3_); Δ_1_(*t*) and Δ_2_(*t*) are the uncertainty part and the external disturbance moment, respectively; and |Δ_1_(*t*)| ≤ *ρ*_1_ , |Δ_2_(*t*)| ≤ *ρ*_2_.

The following lemma was introduced to facilitate the observer and controller stability analysis.

**Lemma 1 (see [1]).**

For *V* : [0, *∞*) ∈ *R*, the solution of $\dot{V}\leq -\alpha V+f$ with ∀ *t* ≥ *t*_0_ ≥ 0 can be expressed as an inequality:

(3) $$\begin{array}{c} V\left(t\right)\leq e^{-\alpha \left(t-t_{0}\right)}V\left(t_{0}\right)+\int_{t_{0}}^{t}e^{-\alpha \left(t-\tau \right)}f\left(\tau \right)\text{d}\tau , \end{array}$$

where *a* is an arbitrary constant.

## 3. The Observer and Controller Design

### 3.1. The Observer Design

The observer of *x*_2_ and *x*_4_ was designed as follows.

To realize *x*_2_ and *x*_4_ observations, the following reconfiguration system was developed:

(4) $$\begin{array}{c} \left\{\begin{array}{c} {\dot{\lambda }}_{1}=\lambda_{2}+l_{1}\left(x_{1}-\lambda_{1}\right)+D_{1}\left(x_{1}-\lambda_{1}\right),\\ {\dot{\lambda }}_{2}=a_{1}x_{3}+f_{1}\left(x_{1}\right)+{\bar{D}}_{2}\left(x_{1}-\lambda_{1}\right),\\ {\dot{\lambda }}_{3}=\lambda_{1}+l_{2}\left(x_{3}-\lambda_{3}\right)+D_{3}\left(x_{3}-\lambda_{3}\right),\\ {\dot{\lambda }}_{4}=a_{2}u+f_{2}\left(x_{1},x_{3}\right)+{\bar{D}}_{4}\left(x_{3}-\lambda_{3}\right), \end{array}\right) \end{array}$$

where *l*_1_, *l*_2_, *D*_1_, ${\bar{D}}_{2}$, *D*_3_, and ${\bar{D}}_{4}$ are the positive real numbers to be designed and *λ*_1_, *λ*_2_, *λ*_3_, and *λ*_4_ are meaningless intermediate state variables.

Then, the observer was designed as

(5) $$\begin{array}{c} \left\{\begin{array}{c} {\hat{x}}_{1}=\lambda_{1},\\ {\hat{x}}_{2}=\lambda_{2}+l_{1}\left(x_{1}-\lambda_{1}\right),\\ {\hat{x}}_{3}=\lambda_{3},\\ {\hat{x}}_{4}=\lambda_{4}+l_{2}\left(x_{3}-\lambda_{3}\right), \end{array}\right) \end{array}$$

where ${\hat{x}}_{i}$ is the state estimation. The estimation error can be defined as

(6) $$\begin{array}{c} {\tilde{x}}_{i}=x_{i}-{\hat{x}}_{i}. \end{array}$$

From equations (4)–(6), we have

(7) $$\begin{array}{c} \left\{\begin{array}{c} {\dot{\hat{x}}}_{1}=\lambda_{2}+l_{1}\left(x_{1}-\lambda_{1}\right)+D_{1}\left(x_{1}-\lambda_{1}\right)={\hat{x}}_{2}+D_{1}{\tilde{x}}_{1},\\ {\dot{\hat{x}}}_{2}=a_{1}x_{3}+f_{1}\left(x_{1}\right)+{\bar{D}}_{2}\left(x_{1}-\lambda_{1}\right)+l_{1}\left(x_{2}-{\hat{x}}_{2}-D_{1}{\tilde{x}}_{1}\right)\\ =a_{1}x_{3}+f_{1}\left(x_{1}\right)+l_{1}{\tilde{x}}_{2}+\left({\bar{D}}_{2}-l_{1}D_{1}\right){\tilde{x}}_{1},\\ {\dot{\hat{x}}}_{3}=\lambda_{4}+l_{2}\left(x_{3}-\lambda_{3}\right)+D_{3}\left(x_{3}-\lambda_{3}\right)={\hat{x}}_{4}+D_{3}{\tilde{x}}_{3},\\ {\dot{\hat{x}}}_{4}=a_{2}u+f_{2}\left(x_{1},x_{3}\right)+{\bar{D}}_{4}\left(x_{3}-\lambda_{3}\right)+l_{2}\left(x_{4}-{\hat{x}}_{4}-D_{3}{\tilde{x}}_{3}\right)\\ =a_{2}u+f_{2}\left(x_{1},x_{3}\right)+l_{2}{\tilde{x}}_{4}+\left({\bar{D}}_{4}-l_{2}D_{3}\right){\tilde{x}}_{3}. \end{array}\right) \end{array}$$

Note that $D_{2}={\bar{D}}_{2}-l_{1}D_{1}$ and $D_{4}={\bar{D}}_{4}-l_{2}D_{3}$. Then,

(8) $$\begin{array}{c} \left\{\begin{array}{c} {\dot{\hat{x}}}_{1}={\hat{x}}_{2}+D_{1}{\tilde{x}}_{1},\\ {\dot{\hat{x}}}_{2}=a_{1}x_{3}+f_{1}\left(x_{1}\right)+l_{1}{\tilde{x}}_{2}+D_{2}{\tilde{x}}_{1},\\ {\dot{\hat{x}}}_{3}={\hat{x}}_{4}+D_{3}{\tilde{x}}_{3},\\ {\dot{\hat{x}}}_{4}=a_{2}u+f_{2}\left(x_{1},x_{3}\right)+l_{2}{\tilde{x}}_{4}+D_{4}{\tilde{x}}_{3}. \end{array}\right) \end{array}$$

The following theorem was introduced to facilitate the proof of observer convergence.

**Theorem 1 .**

For system (2) and observer (5), if the initial conditions satisfy *V*(0) ≤ *p*, where *p* is any positive real number, there exists a condition that all the signals *l*_1_, *l*_2_, *D*_*i*_(*i*=1,…, 4) of the system are semiglobally consistent and bounded, and the observation error converges to an arbitrarily small residual set.

**Proof**

According to equations (5) and (6), the Lyapunov function is taken as

(9) $$\begin{array}{c} V=\frac{1}{2}\sum_{i=1}^{4}{\tilde{x}}_{i}^{2}. \end{array}$$

The following can be derived from equation (9):

(10) $$\begin{array}{c} \dot{V}={\tilde{x}}_{1}\left(x_{2}-{\hat{x}}_{2}-D_{1}{\tilde{x}}_{1}\right)+{\tilde{x}}_{2}\left(\Delta_{1}-l_{1}{\tilde{x}}_{2}-D_{2}{\tilde{x}}_{1}\right)+{\tilde{x}}_{3}\left(x_{4}-{\hat{x}}_{1}-D_{3}{\tilde{x}}_{3}\right)+{\tilde{x}}_{4}\left(\Delta_{2}-l_{2}{\tilde{x}}_{4}-D_{1}{\bar{x}}_{3}\right)\\ =\left(1-D_{2}\right){\tilde{x}}_{1}{\tilde{x}}_{2}+\left(1-D_{4}\right){\tilde{x}}_{3}{\tilde{x}}_{4}-D_{1}{\tilde{x}}_{1}^{2}-l_{1}{\tilde{x}}_{2}^{2}-D_{3}{\tilde{x}}_{3}^{2}-l_{2}{\tilde{x}}_{4}^{2}+\Delta_{1}{\tilde{x}}_{2}+\Delta_{2}{\tilde{x}}_{4}. \end{array}$$

Taking *D*_2_=*D*_1_=1 and the inequality $\rho_{i}^{2}/2+{\tilde{x}}_{j}^{2}/2\geq \rho_{i\;}$, $\left|{\tilde{x}}_{j}\right|\geq \Delta_{i}{\tilde{x}}_{i}$, we have

(11) $$\begin{array}{c} \dot{V}\leq -D_{1}{\tilde{x}}_{1}^{2}-l_{1}{\tilde{x}}_{2}^{2}-D_{3}{\tilde{x}}_{3}^{2}-l_{2}{\tilde{x}}_{4}^{2}+\frac{\rho_{1}^{2}}{2}+\frac{{\tilde{x}}_{2}^{2}}{2}+\frac{\rho_{2}^{2}}{2}+\frac{{\tilde{x}}_{4}^{2}}{2}. \end{array}$$

Inequality (11) can be rectified as

(12) $$\begin{array}{c} \dot{V}\leq -\left(D_{1}{\tilde{x}}_{1}^{2}+D_{3}{\tilde{x}}_{3}^{2}+\left(l_{1}-\frac{1}{2}\right){\tilde{x}}_{2}^{2}+\left(l_{2}-\frac{1}{2}\right){\tilde{x}}_{4}^{2}\right)+\frac{\rho_{1}^{2}}{2}+\frac{\rho_{2}^{2}}{2}. \end{array}$$

Taking *l*_1_ ≥ (1/2)+*r*, *l*_2_ ≥ (1/2)+*r*, *D*_1_ ≥ *r*, and *D*_3_ ≥ *r* with *r* being the positive real number to be designed,

(13) $$\begin{array}{c} D_{1}{\tilde{x}}_{1}^{2}+D_{3}{\tilde{x}}_{3}^{2}+\left(l_{1}-\frac{1}{2}\right){\tilde{x}}_{2}^{2}+\left(l_{2}-\frac{1}{2}\right){\tilde{x}}_{4}^{2}\geq r\left({\tilde{x}}_{1}^{2}+{\tilde{x}}_{3}^{2}+{\tilde{x}}_{2}^{2}+{\tilde{x}}_{4}^{2}\right). \end{array}$$

Thus,

(14) $$\begin{array}{c} \dot{V}\leq -r\left({\tilde{x}}_{1}^{2}+x_{3}^{2}+{\tilde{x}}_{2}^{2}+{\tilde{x}}_{4}^{2}\right)+\frac{\rho_{1}^{2}}{2}+\frac{\rho_{2}^{2}}{2}\leq -2rV+Q, \end{array}$$

where *Q*=*ρ*_1_^2^/2+*ρ*_2_^2^/2.

According to Lemma 1, the solution to inequality (14) is

(15) $$\begin{array}{c} V\left(t\right)\leq e^{-2r\left(t-t_{0}\right)}V\left(t_{0}\right)+Qe^{-2rt}\int_{t_{0}}^{t}e^{2r\tau }\text{d}\tau =e^{-2r\left(t-t_{0}\right)}V\left(t_{0}\right)+\frac{Qe^{-2rt}}{2r}\left(e^{2rt}-e^{2rt_{0}}\right)=e^{-2r\left(t-t_{0}\right)}V\left(t_{0}\right)+\frac{Q}{2r}\left(1-e^{-2r\left(t-t_{0}\right)}\right). \end{array}$$

That is,

(16) $$\begin{array}{c} V\left(t\right)\leq \frac{Q}{2r}+\left(V\left(t_{0}\right)-\frac{Q}{2r}\right)e^{-2r\left(t-t_{0}\right)}. \end{array}$$

Then, all the signals of the system are semiglobally bounded and satisfy

(17) $$\begin{array}{c} \underset{t⟶\infty }{\lim}V\left(t\right)\leq \frac{Q}{2r}. \end{array}$$

**Remark 1 .**

From equation (17), it can be inferred that the observation accuracy of the state depends on the upper bound Δ_1_(*t*) and the initial error Δ_2_(*t*) of the observer. When parameter *r* is infinitely large, the observation error will be arbitrarily small.

**Remark 2 .**

Without considering the modelling uncertainty Δ_1_(*t*)=0 and the external disturbance moment Δ_2_(*t*)=0, (*ρ*_1_^2^/2)+(*ρ*_2_^2^/2)=0, that is, if $\dot{V}\leq -2rV$, then *V*(*t*) ≤ *e*^−2*r*(*t* − *t*_0_)^*V*(*t*_0_). At this point, the observer converges exponentially.

### 3.2. Design and Analysis of Observer-Based Sliding Mode Controller

Observer-based sliding mode control is a new sliding mode control method in recent years. It solves the unknown disturbance problem directly from the sliding mode design side by purposefully designing the switching function and realizes the global nonsingular control of the system. At the same time, it inherits the finite-time convergence characteristics of sliding mode. Compared with the traditional sliding mode control, it can make the control system converge to the desired trajectory in finite time and has high steady-state accuracy. It is especially suitable for high-speed and high-precision control.

Let *x*_1_ and *x*_2_ be the controlled targets of *x*_*d*_ and ${\dot{x}}_{d}$, respectively. The design error can be expressed as

(18) $$\begin{array}{c} \left\{\begin{array}{c} e_{1}=x_{1}-x_{d},\\ e_{2}={\dot{e}}_{1}=x_{2}-{\dot{x}}_{d},\\ e_{3}={\ddot{e}}_{1}={\dot{x}}_{2}-{\ddot{x}}_{d}=a_{1}x_{3}+f_{1}\left(x_{1}\right)-{\ddot{x}}_{d},\\ e_{4}={\ddot{e}}_{1}=a_{1}{\dot{x}}_{3}+{\dot{f}}_{1}\left(x_{1}\right)-{\dddot{x}}_{d}=a_{1}x_{4}+{\dot{f}}_{1}\left(x_{1}\right)-{\dddot{x}}_{d}. \end{array}\right) \end{array}$$

Then, the error of the observer can be expressed as

(19) $$\begin{array}{c} \left\{\begin{array}{c} {\hat{e}}_{1}={\hat{x}}_{1}-x_{d},\\ {\hat{e}}_{2}={\hat{x}}_{2}-{\dot{x}}_{d},\\ {\hat{e}}_{3}=a_{1}{\hat{x}}_{3}+{\hat{f}}_{1}\left(x_{1}\right)-{\ddot{x}}_{d},\\ {\hat{e}}_{4}=a_{1}{\hat{x}}_{4}+{\hat{\dot{f}}}_{1}\left(x_{1}\right)-{\dddot{x}}_{d}. \end{array}\right) \end{array}$$

From equations (18) and (19), we have

(20) $$\begin{array}{c} \left\{\begin{array}{c} {\tilde{e}}_{1}=e_{1}-{\hat{e}}_{1}={\tilde{x}}_{1},\\ {\tilde{e}}_{2}=e_{2}-{\hat{e}}_{2}={\tilde{x}}_{2},\\ {\tilde{e}}_{3}=e_{3}-{\hat{e}}_{3}=a_{1}{\tilde{x}}_{3}+f_{1}\left(x_{1}\right)-{\hat{f}}_{1}\left(x_{1}\right),\\ {\tilde{e}}_{4}=e_{4}-{\hat{e}}_{4}=a_{1}{\tilde{x}}_{4}+{\dot{f}}_{1}\left(x_{1}\right)-{\hat{\dot{f}}}_{1}\left(x_{1}\right). \end{array}\right) \end{array}$$

The design sliding mode function can be expressed as

(21) $$\begin{array}{c} s=c_{1}e_{1}+c_{2}e_{2}+c_{3}e_{3}+e_{4}, \end{array}$$

where *c*_*i*_ > 0 is designed by *i*=1,2,3.

Then,

(22) $$\begin{array}{c} \hat{s}=c_{1}{\tilde{e}}_{1}+c_{2}{\tilde{e}}_{2}+c_{3}{\tilde{e}}_{3}+{\tilde{e}}_{4}=c_{1}{\tilde{x}}_{1}+c_{2}{\tilde{x}}_{2}+c_{3}\left(a_{1}{\tilde{x}}_{3}+f_{1}\left(x_{1}\right)-{\hat{f}}_{1}\left(x_{1}\right)\right)+a_{1}{\tilde{x}}_{4}+{\dot{f}}_{1}\left(x_{1}\right)-{\hat{\dot{f}}}_{1}\left(x_{1}\right). \end{array}$$

Then, the control law can be designed as

(23) $$\begin{array}{c} u=-\frac{1}{a_{1}a_{2}}\left[c_{1}\left({\hat{x}}_{2}-{\dot{x}}_{d}\right)+c_{2}\left(a_{1}{\hat{x}}_{3}+{\hat{f}}_{1}\left(x_{1}\right)-{\ddot{x}}_{d}\right)+c_{3}\left(a_{1}{\hat{x}}_{4}+{\hat{\dot{f}}}_{1}\left(x_{1}\right)-{\dddot{x}}_{d}\right)+a_{1}{\hat{f}}_{1}\left(x_{1},x_{3}\right)+\hat{{\ddot{f}}_{1}}\left(x_{1}\right)-{\dddot{x}}_{d}+\eta \hat{s}\right], \end{array}$$

where *η* > 0.

Then, we have

(24) $$\begin{array}{c} \dot{s}=c_{1}{\dot{e}}_{1}+c_{2}{\dot{e}}_{2}+c_{3}{\dot{e}}_{3}+{\dot{e}}_{1}\\ =c_{1}\left(x_{2}-{\dot{x}}_{d}\right)+c_{2}\left(a_{1}x_{3}+f_{1}\left(x_{1}\right)-{\overset{¨}{x}}_{d}\right)+c_{3}\left(a_{1}x_{4}+{\dot{f}}_{1}\left(x_{1}\right)-{\dddot{x}}_{d}\right)+a_{1}\left(a_{2}u+f_{1}\left(x_{1},x_{3}\right)\right)+{\ddot{f}}_{1}\left(x_{1}\right)-{\dddot{x}}_{d}\\ =c_{1}\left(x_{2}-{\dot{x}}_{d}\right)+c_{2}\left(a_{1}x_{3}+f_{1}\left(x_{1}\right)-{\ddot{x}}_{d}\right)+c_{3}\left(a_{1}x_{4}+{\dot{f}}_{1}\left(x_{1}\right)-{\dddot{x}}_{d}\right)\\ -\left[c_{1}\left({\hat{x}}_{2}-{\dot{x}}_{d}\right)+c_{2}\left(a_{1}{\hat{x}}_{3}+{\hat{f}}_{1}\left(x_{1}\right)-{\ddot{x}}_{d}\right)+c_{3}\left(a_{1}{\hat{x}}_{4}+{\hat{\dot{f}}}_{1}\left(x_{1}\right)-{\dddot{x}}_{d}\right)+a_{1}{\hat{f}}_{1}\left(x_{1},x_{3}\right)+{\hat{f}}_{1}\left(x_{1}\right)-{\dddot{x}}_{d}+\eta \hat{s}\right]\\ +a_{1}f_{1}\left(x_{1},x_{3}\right)+{\ddot{f}}_{1}\left(x_{1}\right)-{\ddddot{x}}_{d}\\ =c_{1}{\tilde{x}}_{2}+c_{2}a_{1}{\tilde{x}}_{3}+c_{3}a_{1}{\tilde{x}}_{4}+c_{2}\left(f_{1}\left(x_{1}\right)-{\hat{f}}_{1}\left(x_{1}\right)\right)\\ +c_{3}\left({\dot{f}}_{1}\left(x_{1}\right)-{\hat{\dot{f}}}_{1}\left(x_{1}\right)\right)+a_{1}\left(f_{1}\left(x_{1},x_{3}\right)-{\hat{f}}_{1}\left(x_{1},x_{3}\right)\right)+\left({\ddot{f}}_{1}\left(x_{1}\right)-\hat{{\ddot{f}}_{1}}\left(x_{1}\right)\right)-\eta \left(s-\tilde{s}\right). \end{array}$$

Take the Lyapunov function as

(25) $$\begin{array}{c} V_{c}=\frac{1}{2}s^{2}. \end{array}$$

Then,

(26) $$\begin{array}{c} {\dot{V}}_{c}=s\dot{s}=s\left[c_{1}{\tilde{x}}_{2}+c_{2}a_{1}{\tilde{x}}_{3}+c_{3}a_{1}{\tilde{x}}_{4}+c_{2}\left(f_{1}\left(x_{1}\right)-{\hat{f}}_{1}\left(x_{1}\right)\right)+c_{3}\left({\dot{f}}_{1}\left(x_{1}\right)-{\hat{\dot{f}}}_{1}\left(x_{1}\right)\right)\right.\\ +a_{1}\left(f_{1}\left(x_{1},x_{3}\right)-{\hat{f}}_{1}\left(x_{1},x_{3}\right)\right)+\left({\ddot{f}}_{1}\left(x_{1}\right)-\hat{{\ddot{f}}_{1}}\left(x_{1}\right)\right)-\eta \left(s-\tilde{s}\right)\\ =-\eta s^{2}+\eta s\left(c_{1}{\tilde{x}}_{1}+c_{2}{\tilde{x}}_{2}+c_{3}\left(a_{1}{\tilde{x}}_{3}+f_{1}\left(x_{1}\right)-{\hat{f}}_{1}\left(x_{1}\right)\right)+a_{1}{\tilde{x}}_{4}+{\dot{f}}_{1}\left(x_{1}\right)-{\hat{\dot{f}}}_{1}\left(x_{1}\right)\right)\\ +s\left[c_{1}{\tilde{x}}_{2}+c_{2}a_{1}{\tilde{x}}_{3}+c_{3}a_{1}{\tilde{x}}_{4}+c_{2}\left(f_{1}\left(x_{1}\right)-{\hat{f}}_{1}\left(x_{1}\right)\right)+c_{3}\left({\dot{f}}_{1}\left(x_{1}\right)-{\hat{\dot{f}}}_{1}\left(x_{1}\right)\right)\right.\\ +a_{1}\left(f_{1}\left(x_{1},x_{3}\right)-{\hat{f}}_{1}\left(x_{1},x_{3}\right)\right)+\left({\ddot{f}}_{1}\left(x_{1}\right)-\hat{{\ddot{f}}_{1}}\left(x_{1}\right)\right)\left(\right]\\ =-\eta s^{2}+s\left[\eta c_{1}{\tilde{x}}_{1}+\left(\eta c_{2}+c_{1}\right){\tilde{x}}_{2}+\left(\eta c_{3}a_{1}+c_{2}a_{1}\right){\tilde{x}}_{3}+\left(\eta a_{1}+c_{3}a_{1}\right){\tilde{x}}_{4}\right.\\ +\left(\eta c_{3}+c_{2}\right)\left(f_{1}\left(x_{1}\right)-{\hat{f}}_{1}\left(x_{1}\right)\right)+\left(\eta +c_{3}\right)\left({\dot{f}}_{1}\left(x_{1}\right)-{\hat{\dot{f}}}_{1}\left(x_{1}\right)\right)\\ +a_{1}\left(f_{1}\left(x_{1},x_{3}\right)-{\hat{f}}_{1}\left(x_{1},x_{3}\right)\right)+\left({\ddot{f}}_{1}\left(x_{1}\right)-\hat{{\ddot{f}}_{1}}\left(x_{1}\right)\right)\left(\right]\\ =-\eta s^{2}+s\chi \left(\tilde{x}\right)\leq -\eta s^{2}+\frac{1}{2}s^{2}+\frac{1}{2}\chi^{2}\left(\tilde{x}\right)\\ =\left(\frac{1}{2}-\eta \right)s^{2}+\frac{1}{2}\chi^{2}\left(\tilde{x}\right)=\left(1-2\eta \right)V_{c}+\frac{1}{2}\chi^{2}\left(\tilde{x}\right), \end{array}$$

where

(27) $$\begin{array}{c} \chi \left(\tilde{x}\right)=\left[\eta c_{1}{\tilde{x}}_{1}+\left(\eta c_{2}+c_{1}\right){\tilde{x}}_{2}+\left(\eta c_{3}a_{1}+c_{2}a_{1}\right){\tilde{x}}_{3}+\left(\eta a_{1}+c_{3}a_{1}\right){\tilde{x}}_{1}\right.\\ +\left(\eta c_{3}+c_{2}\right)\left(f_{1}\left(x_{1}\right)-{\hat{f}}_{1}\left(x_{1}\right)\right)+\left(\eta +c_{3}\right)\left({\dot{f}}_{1}\left(x_{1}\right)-{\hat{\dot{f}}}_{1}\left(x_{1}\right)\right)\\ +a_{1}\left(f_{1}\left(x_{1},x_{3}\right)-{\hat{f}}_{1}\left(x_{1},x_{3}\right)\right)+{\ddot{f}}_{1}\left(x_{1}\right)-\hat{{\ddot{f}}_{1}}\left(x_{1}\right)\left(\right]. \end{array}$$

Since observer (5) converges exponentially, i.e., at time *t*⟶*∞*, ${\tilde{x}}_{1}$ converges exponentially to ${\tilde{x}}_{2}$, and ${\tilde{x}}_{3}$ to ${\tilde{x}}_{4}$. According to the Taylor series expansion of *f*_1_(*x*_1_)=−*Mgl*/*I* · sin  *x*_1_ − *K*/*I* · *x*_1_ and *f*_2_(*x*_1_, *x*_3_)=*K*/*J* · (*x*_1_ − *x*_3_), $f_{1}\left(x_{1}\right)⟶{\hat{f}}_{1}\left(x_{1}\right)$ converges exponentially to ${\dot{f}}_{1}\left(x_{1}\right)⟶{\hat{\dot{f}}}_{1}\left(x_{1}\right)$, $f_{1}\left(x_{1},x_{3}\right)⟶{\hat{f}}_{1}\left(x_{1},x_{3}\right)$. Thus, ${\ddot{f}}_{1}\left(x_{1}\right)⟶\hat{{\ddot{f}}_{1}}\left(x_{1}\right)$ also converges exponentially to 0.

Considering the observer and the controller, the Lyapunov function of the closed loop is taken as

(28) $$\begin{array}{c} V=V_{c}+V_{o}. \end{array}$$

According to equation (28), we have

(29) $$\begin{array}{c} \dot{V}={\dot{V}}_{0}+{\dot{V}}_{c}\leq -2rV_{0}-\left(2\eta -1\right)V_{c}+\frac{1}{2}\chi^{2}\left(\tilde{x}\right)\leq -\eta_{1}V+\chi \left(\cdot \right)e^{-\sigma_{0}\left(t-t_{0}\right)}, \end{array}$$

where *η*_1_={2*r*, (2*η* − 1)}_max_; *χ*(·) is the class *K* function of $\left\|\tilde{x}\left(t_{0}\right)\right\|$; and *σ*_0_ > 0.

According to Lemma 1, the solution to $\dot{V}\leq -\eta_{1}V+\chi \left(\cdot \right)e^{-\sigma_{0}\left(t-t_{0}\right)}$ can be expressed as an inequality:

(30) $$\begin{array}{c} V\left(t\right)\leq e^{-\eta_{1}\left(t-t_{0}\right)}V\left(t_{0}\right)+\chi \left(\Delta \right)\int_{t_{0}}^{t}e^{-\eta_{1}\left(t-\tau \right)}e^{-\sigma_{0}\left(\tau -t_{0}\right)}\text{d}\tau \\ =e^{-\eta_{1}\left(t-t_{0}\right)}V\left(t_{0}\right)+\chi \left(\cdot \right)e^{-\eta_{1}t+\sigma_{0}t_{0}}\int_{t_{0}}^{t}e_{1}^{\eta_{1}\tau }e^{-\sigma_{0}\tau }\text{d}\tau \\ =e^{-\eta_{1}\left(t-t_{0}\right)}V\left(t_{0}\right)+{\frac{\chi \left(\Delta \right)}{\eta_{1}-\sigma_{0}}e^{-\eta_{1}t+\sigma_{0}t_{0}}e^{\left(\eta_{1}-\sigma_{0}\right)\tau }|}_{t_{0}}^{t}\\ =e^{-\eta_{1}\left(t-t_{0}\right)}V\left(t_{0}\right)+\frac{\chi \left(\Delta \right)}{\eta_{1}-\sigma_{0}}e^{-\eta_{1}t+\sigma_{0}t_{0}}\left(e^{\left(\eta_{1}-\sigma_{0}\right)t}-e^{\left(\eta_{1}-\sigma_{0}\right)t_{0}}\right)\\ =e^{-\eta_{1}\left(t-t_{0}\right)}V\left(t_{0}\right)+\frac{\chi \left(\cdot \right)}{\eta_{1}-\sigma_{0}}\left(e^{-\sigma_{0}\left(t-t_{0}\right)}-e^{-\eta_{1}\left(t-t_{0}\right)}\right). \end{array}$$

That is, lim_*t*⟶*∞*_*V*(*t*) ≤ 0.

Since *V*(*t*) ≥ 0, when *t*⟶*∞*, *V*(*t*)=0, and *V*(*t*) converges exponentially. The convergence accuracy depends on *η*_1_, i.e., *r* and *η*.

**Remark 3 .**

When the controller reaches the sliding mode surface, that is, *s*=0, we have *e*_4_=−*c*_1_*e*_1_ − *c*_2_*e*_2_ − *c*_3_*e*_3_. If $E_{1}={\left[\begin{array}{ccc} e_{1} & e_{2} & e_{3} \end{array}\right]}^{T}$ and $A=\left[\begin{array}{ccc} 0 & 1 & 0\\ 0 & 0 & 1\\ -c_{1} & -c_{2} & -c_{3} \end{array}\right]$, then ${\dot{E}}_{1}=\;AE_{1}$. Through the design of *c*_1_, *c*_2_, and *c*_3_, *A* is Hurwitz zeta function. Thus, at time $t⟶\infty ,E_{1}={\left[\begin{array}{ccc} e_{1} & e_{2} & e_{3} \end{array}\right]}^{T}⟶0$. To make *A* as a Hurwitz zeta function, the real root part of the following equation must be negative:

(31) $$\begin{array}{c} \left|A-\lambda I\right|=\left|\begin{array}{ccc} -\lambda & 1 & 0\\ 0 & -\lambda & 1\\ -c_{1}-c_{2} & -c_{3}-\lambda & \; \end{array}\right|=\lambda^{2}\left(-c_{3}-\lambda \right)-c_{1}-c_{2}\lambda . \end{array}$$

That is, −*λ*^3^ − *c*_3_*λ*^2^ − *c*_2_*λ* − *c*_1_=0. Taking the eigenvalue of −10, (*λ*+10)^3^=0, from *λ*^3^+9*λ*^2^+27*λ*+27=0, we can obtain that *λ*^3^+*c*_3_*λ*^2^+*c*_2_*λ*+*c*_1_=0, *c*_1_=1000, *c*_2_=300, and *c*_3_=30. Hence, the convergence condition can be satisfied.

## 4. Results and Discussion

### 4.1. The Simulation of the Observer

To verify the feasibility of the robust observer, a system was developed to run in an open loop and modelled considering the following external disturbance moments and modelling uncertainties:

(32) $$\begin{array}{c} \left\{\begin{array}{c} {\dot{\theta }}_{1}=\omega_{1},\\ {\dot{\omega }}_{1}=a_{1}\theta_{m}+f_{1}\left(\theta_{1}\right)+\Delta_{1}\left(t\right),\\ {\dot{\theta }}_{m}=\omega_{m},\\ {\dot{\omega }}_{m}=a_{2}u+f_{2}\left(\theta_{1},\theta_{m}\right)+\Delta_{2}\left(t\right), \end{array}\right) \end{array}$$

where *θ*_1_, *ω*_1_, *θ*_*m*_, and *ω*_*m*_ are the position of rod 1, the angular velocity of rod 1, the position of rod *m*, and the angular velocity of rod *m*, respectively. The parameters were configured as follows: *x*=[*θ*_1_*ω*_1_,…,*θ*_*m*_*ω*_*m*_]^*T*^, Δ_1_(*t*)=sin  *t*, Δ_2_(*t*)=cos  *t*, *J*=1 kg · m^2^, *Mgl*=5 Nm, and *K*=40 Nm/rad. Before simulation, the system state was initialized as $x\left(0\right)={\left[\begin{array}{cccc} 0.1 & 0 & 0.05 & 0 \end{array}\right]}^{T}$, and the observer state is initialized as $\lambda \left(0\right)={\left[\begin{array}{cccc} 0 & 0 & 0 & 0 \end{array}\right]}^{T}$. The observer adopts the form of (4) and (5), with *r*=100. Based on *l*_1_ ≥ 1/2+*r* (5), *l*_2_ ≥ 1/2+*r*, *D*_1_ ≥ *r*, and *D*_2_ ≥ *r*, the following parameter values were selected: *l*_1_=*l*_2_=101, *D*_2_=*D*_4_=1.0, and *D*_1_=*D*_3_=101.

The simulation structure of the observer is given in Figure 1, and the simulation results are shown in Figures 2 and 3. Specifically, Figure 2 presents the flexible modes of the position states of the two joints and their derivatives (i.e., velocities), and Figure 3 displays the tracking errors of the states. It can be inferred that the proposed observer can completely observe each state of the system (as suggested by Figure 2) and fully track the states of the upper two joints after only 0.1 s (as indicated by the error curve in Figure 3, the errors are 0.001, 0.15, 0.0015, and 0.12 for Figures 3(a)–3(d)). Therefore, our method was proved to be fast and effective. Although there are disturbances in the system, i.e., Δ_1_(*t*)=sin  *t* and Δ_2_(*t*)=cos  *t*, the observation results show the anti-interference ability and good robustness of the proposed observer.

### 4.2. The Simulation of the Control Algorithm

To verify the effectiveness of the proposed control algorithm, the system with Δ_1_(*t*)=0.15  sin  *t* and Δ_2_(*t*)=0.23  cos  *t* was taken as shown in equation (32), where $x\left(0\right)={\left[\begin{array}{cccc} 0.2 & 0 & 0 & 0 \end{array}\right]}^{T}$ and disturbance torque is $\lambda \left(0\right)={\left[\begin{array}{cccc} 0 & 0 & 0 & 0 \end{array}\right]}^{T}$. The other parameters were kept the same as in simulation 1. The controller takes equation (23), with *c*_1_=1000, *c*_2_=300, *c*_3_=30, and *η*=1.5. The desired trajectory of joint 2 is *θ*_1  *d*_=sin. The simulation results are shown in Figures 4 and 5. The former presents the angle and angular velocity of the second joint of the manipulator, and the latter exhibits the observed values of each state of the manipulator.

As shown in Figure 4, the system state was stabilized in a limited time, despite the presence of external disturbances and fault signals, indicating that the system converges well under this controller. Because the initial state of the system is $x\left(0\right)={\left[\begin{array}{cccc} 0.2 & 0 & 0 & 0 \end{array}\right]}^{T}$ and due to the existence of interference, there is a large error at the initial time. However, with the increase of control time, the system error decreases rapidly. Hence, our control method can effectively deal with the above problem.  Figure 5 shows the results with PID controller; it can be seen that there is a large error in the position of PID control, and especially when the position reaches the maximum and minimum, the error is large.

As shown in Figure 6, our disturbance observer could observe the state information of the system with high accuracy and effectiveness. That is, the observed signals can be used in the controller design, which further illustrates the effectiveness of the method.

## 5. Conclusions

The improvement of a robust observer-based sliding mode is improved, and the efficiency of the model is improved in this paper. Aiming at the problems of high nonlinearity, strong coupling, and external interference in the system, we firstly designed a state observer for the system through the auxiliary reconstruction system, solved the state observation problem of the system, clarified the convergence condition of the observer through theoretical analysis, and verified it through simulation. Then, the position and velocity tracking problem was tackled. Considering the external disturbance, a sliding mode control of the flexible-joint manipulator was derived based on the robust observer. The control method ensures that the system state can converge exponentially to zero in finite time under different inputs and outputs. The simulation results show that the observer can quickly observe the state variables of the system. Also, combined with the sliding mode controller, the system error can quickly converge to zero. The proposed control strategy is simple and easy to implement.

## Figures and Tables

**Figure 1:** Simulation structure of the observer.

**Figure 2:** State estimations. (a) *θ* state estimation. (b) *ω* state estimation. (c) *θ*_*m*_ state estimation. (d) *ω*_*m*_ state estimation.

**Figure 3:** State estimation errors. (a) *θ* estimation error. (b) *ω* estimation error. (c) *θ*_*m*_ estimation error. (d) *ω*_*m*_ estimation error.

**Figure 4:** Angle and angular velocity tracking with the proposed method. (a) Angle tracking. (b) Angular velocity tracking.

**Figure 5:** Angle and angular velocity tracking with PID control. (a) Angle tracking. (b) Angular velocity tracking.

**Figure 6:** Observation of each state of the manipulator.

## Data Availability

The data used to support the findings of this study are available from the corresponding author upon request.
